RETRACTED

# Effect of Riluzole on the Expression of HCN2 in Dorsal Root Ganglion Neurons of Diabetic Neuropathic Pain Rats

**DOI:** 10.1155/2022/8313415

**Published:** 2022-04-06

**Authors:** Dong-mei Zhou, Feng-Jie Shen, Rong Hao, Bei-Miao, Jin-Kui Yang

**Affiliations:** ^1^Department of Endocrinology, Beijing Tongren Hospital, Capital Medical University, Beijing 100730, China; ^2^Department of Endocrinology, Affiliated Hospital of Xuzhou Medical University, Xuzhou 221000, China; ^3^Department of Gastroenterology, Affiliated Hospital of Xuzhou Medical University, Xuzhou 221000, China; ^4^Peixian People's Hospital, Xuzhou 221600, China

## Abstract

Neuropathic pain since early diabetes swamps patients' lives, and diabetes mellitus has become an increasingly worldwide epidemic. No agent, so far, can terminate the ongoing diabetes. Therefore, strategies that delay the process and the further complications are preferred, such as diabetic neuropathic pain (DNP). Dysfunction of ion channels is generally accepted as the central mechanism of diabetic associated neuropathy, of which hyperpolarization-activated cyclic nucleotide-gated 2 (HCN2) ion channel has been verified the involvement of neuropathic pain in dorsal root ganglion (DRG) neurons. Riluzole is a benzothiazole compound with neuroprotective properties on intervention to various ion channels, including hyperpolarization-activated voltage-dependent channels. To investigate the effect of riluzole within lumbar (L3-5) DRG neurons from DNP models, streptozocin (STZ, 70 mg/kg) injection was recruited subcutaneously followed by paw withdrawal mechanical threshold (PWMT) and paw withdrawal thermal latency (PWTL), which both show significant reduction, whilst relieved by riluzole (4 mg/kg/d) administration, which was performed once daily for 7 consecutive days for 14 days. HCN2 expression was also decreased in line with alleviated behavioral tests. Our results indicate riluzole as the alleviator to STZ-induced DNP with involvement of downregulated HCN2 in lumbar DRG by continual systemic administration in rats.

## 1. Introduction

Diabetic neuropathic pain (DNP) is the most common complication in patients with early diabetes mellitus associated neuropathy. People around the world suffer from hyperalgesia and abnormal pain [1–4]. Unfortunately, there are no processing-terminable treatments for diabetic neuropathy (DN) other than improved lifestyle and diabetes control [5, 6], despite the limited prevention in type 1 diabetic patients and the poorly unanimous benefit in type 2 diabetic patients [5, 7, 8]. Therefore, to fail-defended patients, strategies naturally turn to snail the ongoing DN.

Symptoms may emerge early in peripheral nervous system, even during prediabetic stage, which is partially due to poor protection from blood-brain barrier [2]. The primary sensory neurons which function as the connecter between peripheral sensor and central nervous system [9] play an increasingly fundamental role in the generation of neuropathic pain [2, 10]. However, the underlining mechanism is still not fully apprehended. Hyperpolarization-activated, cyclic nucleotide-gated (HCN) channels have been reported to be important members of the voltage-gated pore loop channels family. HCN had unique features by opening at hyperpolarizing potential, carry a Na/K current, and are then regulated by cyclic nucleotides. HCN exert their functions by mediating repetitive action potential firing in the nervous system. The subtype 2 of the hyperpolarization-activated cyclic nucleotide-gated channel family (HCN2) isoform is expressed in nociceptors, and previous studies have suggested that it played a critical role in neuropathic pain. In spite of that, current researches highlight the hyperpolarization-activated cyclic nucleotide-gated 2 (HCN2) ion channel as the crucial driver by modulation of nociceptive afference in rodent DN models of [11–14]. HCN channels are unusual in that they carry an inward current (termed I_*h*_ in neurons) activated time-dependently by hyperpolarization in the range −40 to −140 mV [15], whereas all other voltage-activated channels contrarily being activated by depolarization. Four HCN isoforms, HCN1–4, were cloned in the 1990s [16–18]. They are widely expressed in nervous system, while DRG neurons express HCN isoforms unevenly, of which HCN2 in small-medium neurons [19–23]. Elevations of intracellular cyclic adenosine monophosphate (cAMP) cause a strong shift in the voltage dependence of activation of HCN2 to more positive membrane voltage, causing an increasing I_*h*_ at resting membrane potential [11, 24]. HCN2 channels contribute to the synaptic integration, neuronal excitability, and maintaining the resting membrane potential [15, 19, 25]. Containing majority of the small sensory neurons as nociceptors [21], the present study suggests the involvement of HCN2 ion channel in DNP [11].

RETRACTED

Riluzole is a benzothiazole compound with neuroprotective activities in the treatment of amyotrophic lateral sclerosis [26]. Riluzole has been widely used as the antiglutamate agent for treating the nerve disease amyotrophic lateral sclerosis by changing the activity of substances such as glutamic acid. It has been used for a lone time in clinical practice since 1995, when riluzole was approved by the FDA as the first drug to treat amyotrophic lateral sclerosis. It has been reported that riluzole could block the glutamatergic neurotransmission in the central nervous system, which then lead to neuroprotective effects. In addition to its given clinical applications, recent studies have showed riluzole with increasing evidence of valid antinociceptive properties in various neuropathic pain models, indicating the potential applications in DNP management.

## 2. Materials and Methods

### 2.1. Animals and Materials

The streptozotocin (STZ)-induced diabetic rat model, despite its limitations, is widely applied for type 1 diabetes, in which selective ruin of pancreatic islet *β*-cells triggers insulin deficiency, hyperglycemia, and subsequent DN over several weeks [27, 28]. Hence, we recruited 80 male Sprague-Dawley rats, weighting 200g to 220g (Experimental Animal Center, Xuzhou Medical University), randomly divided into 4 groups (*n* = 20 each): control, DNP, DMSO, and riluzole. For the establishment of diabetic neuropathic pain models, rats underwent subcutaneous injection of STZ (70 mg/kg, Sigma, USA) dissolved in sodium citrate buffer (freshly prepared in ice bath), while those in group control received identical dose of sodium citrate buffer solution. DNP models were successfully prepared with both stable blood glucose from caudal vein measured >16.7 mmol/L on 3 d since STZ injection and the more than 20% declined amplitude of pain threshold measured on 14 d against basic pain threshold. Intraperitoneal injection of riluzole (4 mg/kg/d, Sigma, USA) dissolved in 10%DMSO was given in group riluzole since 14 d to 21 d, while the vehicle alone was injected in group DMSO with the same dose.

### 2.2. Behavioral Test

Paw withdrawal thermal latency (PWTL) and paw withdrawal mechanical threshold (PWMT) targeted on the right hind paw were checked for basal line and remeasured on 3 d, 7 d, 10 d, 14 d, 21 d, and 28 d following SZT injection [29, 30]. For PWTL using IITC series 8 (IITC, USA), rats were primarily placed on a 6 mm-thick glass plate at room temperature (r/*t*). Subsequently, focused heats were approached on the right hind paw, with time recording onset simultaneously. In addition, the reading is justified to 0.01 second. The intensity of heats was modified and the duration was limited within 25 seconds to make rats free from tissue damage. Each rat underwent PWTL 5 times with the same interval of 5 minutes. PWMT was performed with, at most, five trains of von Frey Hairs (Stoelting, USA). The filaments were prepared in arrangement by resulted pressure intensities marked from minimum to maximum. Each stimulus lasted within 4 seconds, whereas a 30-second interval involved. A train got termination till the suffering paw escaping or being licked. Subsequently, the represented pressure was recorded, and the given behaver was labeled as positive. Test was completed for the third positive record. Data were averaged separately for advanced estimation.

RETRACTED

### 2.3. Western Blot

Rats from each group were sacrificed on 21 d, followed by isolation of the L3-5 DRG and storage in liquid nitrogen or at −80°C for subsequent procedures. The frozen DRG were directly homogenized in a lysis buffer containing a cocktail of protease inhibitors. Equal amounts of protein (30 *μ*g) were loaded in each lane and separated by 10% sodium dodecyl sulfate-polyacrylamide gel electrophoresis. The membranes were blocked in 3% bovine serum albumin (BSA) for 2 h and then rinsed thrice in washing buffer for 5 min each. Following sequential incubation overnight at 4°C with rabbit anti-HCN2 (1 : 200, Alomone Labs) and mouse anti-*β*-actin (1 : 1000) primary antibody, the blots were rinsed thrice in washing buffer for 5 min each and incubated for 2 h with AP-conjugated goat antirabbit IgG (1 : 1000, Beyotime Biotechnology, Nantong, China) or goat antimouse secondary antibody IgG (1 : 1000). All western blot analyses were performed at least in triplicate, with parallel results obtained. Squares of the same size from each band were measured for density, with the background subtracted. The expression of *β*-actin was used as a loading control for protein expression. The expression level of the proteins is an average of the densities per band area from each group.

### 2.4. Immunofluorescent Test

On 21 d after STZ injection, rats were anesthetized with pentobarbital sodium and transcardially perfused with normal saline succeeded by 4% paraformaldehyde in 0.1 M phosphate buffer saline (PBS). DRGs from L3-5 were isolated, postfixed overnight in 4% paraformaldehyde in 0.1 M PBS, and cryoprotected in 30% sucrose in 0.1 M PB at 4°C till the tissue sinkage to the bottom of the container. Transverse DRG sections (14 *μ*m) were sliced on a cryostat and mounted serially on slides. To visualize HCN2 channels, immunofluorescence labeling methods were used. Briefly, the sections were rinsed twice with 0.1 M PBS and then incubated with a solution containing 0.3% Triton X-100 and 1% donkey serum albumin for 3 h at r/*t*. The sections were thereafter incubated with anti-HCN2 channel antibodies (1 : 200, rabbit anti-HCN2, Alomone Labs) in PBST for 24 h at 4°C. After three washes with PBST, the sections were further incubated with secondary antibody Alexa Fluor 488 (1 : 200, donkey antirabbit IgG, Invitrogen, USA) for 2 h at r/*t*. The sections were then mounted with antifade medium and stored at 4°C. All images were captured with Olympus FV1000 confocal microscope and processed with Adobe Photoshop software. The negative controls were performed using the same procedure without addition of primary antibody.

RETRACTED

### 2.5. Statistics and Analysis

The data are expressed as the mean ± SD. One-way ANOVA, followed by the Student–Newman–Keuls post hoc test, were adopted in measurements of time courses measured for PWMT and PWTL and of HCN2 expression by western blot and immunofluorescence. *P* < 0.05 was considered statistically significant. All of the tests (including behavior, western blotting, and immunofluorescence) were performed blindly by SPSS16.0 software.

## 3. Results

Measurements of paw withdrawal mechanical threshold (PWMT) and paw withdrawal thermal latency (PWTL) in rats were performed.

We tested the basal point of PWMT and PWTL in all rats, and further data were measured on 3 d, 7 d, 10 d, 14 d, 21 d, and 28 d. Parameters from control showed homogeneity at each time point, which is in line with basal (*P* > 0.05). STZ-treated rats showed both significant reduction via PWTL and PWMT since the first postinjection, which was then kept on declining until the plateau on 14 d by PWTL and on 10 d by PWMT, of which level lower in amplitude more than 20% to baseline, respectively (*P* < 0.05). In the context, pain associated threshold tests can indicate the onset of DNP. Hence, we justified the establishment of DNP models on behavioral change. It was found that the group riluzole showed a rise in PMWT and PTWL at 21 d versus group DMSO, while back to the same level 7 days later, as compared with riluzole (*P* < 0.05). Additionally, there is no significant difference between group DNP and DMSO (*P* > 0.05) (Figure 1). Our data suggest that riluzole treatments can alleviate pain-like behaviors induced by both thermal and mechanical stimuli in DNP rats under continuous administration, but completely invalid following the absence of one week.

### 3.1. Expressions of HCN2 by Western Blot in DNP Rats

We tested the HCN2 expression of DRG tissues by western blot. As shown in Figure 2, the densities of HCN2 in group control were significantly lower than the other three groups, whilst riluzole was significantly lower than group DMSO (*P* < 0.05). Additionally, the densities of actin which recruited as endo-parameter showed good homogeneity (*P* > 0.05). Our data illustrated DRG tissues from DNP rats with upregulated HCN2 expression could be downregulated by riluzole.

### 3.2. Expressions of HCN2 by Immunofluorescent Analysis in DNP Rats

Results of immunofluorescent analysis showed upregulations of HCN2 in group DNP, DMSO, and riluzole compared with control (*P* < 0.05). However, the expressions of HCN2 in DRG in group riluzole were downregulated versus group DMSO (*P* < 0.05). There were no significant differences in expression between group DMSO and DNP (*P* > 0.05; Figure 3). The results further supported that riluzole downregulates DRG HCN2 expression in DNP rats.

RETRACTED

## 4. Discussion

Diabetic neuropathic pain is one of the most frequent complications of diabetes, which restricts patients' lives in misfortune [1–4]. Neuropathic pain is defined as pain caused by a lesion or disease affecting the somatosensory system [31], and the main difference of neuropathic pain to others is the paradoxical combination of sensory loss and pain with or without hypersensitive phenomena to one or several sensory modalities in the painful area [2]. Practically, not all DN patients present painful symptoms. However, key distinguishing feature has been described as whether the patients have increased sensitivity to mechanical and thermal stimuli [32]. Therefore, associated threshold tests are consensually recruited as the diagnostic approach for DNP. In parallel, our data of group DNP showed successive decline since STZ administration to 15 d by PWTL and PWMT, while group control had an approximately horizontal line of containment with basal point (Figures 1(a) and 1(b)). Regrettably, DNP can hardly be cured, owing to the irreversibility of diabetic neuropathy which can neither be fully prevented nor reverted by lowering blood glucose levels [33]. DN insults both central and peripheral nervous system, but it comes earlier in the peripheral even during early stage of diabetes due to the prevention from blood-brain barrier [2]. In peripheral nervous system, dorsal root ganglia contain the primary neurons within sensory pathway. They are activated by a variety of internal and external stimuli which integrated here and then transmitted to the central nervous system [9]. Therefore, dysfunction of DRG will change the pattern of resulted signal transmission to the central and contribute to DNP.

Riluzole is the only drug to prolong survival for amyotrophic lateral sclerosis[26]; however, increasing evidences have shown that riluzole has antinociceptive benefit [12, 34–38]. But the underlying mechanism is still obscure. Otherwise, riluzole was reported modulation on hyperpolarization-activated I_*h*_ by shifting its voltage-dependent activation to more hyperpolarized potentials [39], which indicates the antinociceptive role of riluzole potentially involved with HCN actions.

A classic study suggested that the intensity of a sensation is signaled by the frequency of action potentials in afferent nerve fibers, and this is also true in recognoscibility of pain [40]. Stronger the noxious stimuli input, more the ion channels open, and therefore higher level the action potential frequency generated [14]. As increased ability of response to environmental irritants under painful DN, nerve terminals develop more frequent activation to primary sensory neurons, to wit DRG neurons [2]. Accordingly, DNP DRGs tend to receive more nociceptive input than control even under the same noxious stimuli. By the way, the present data suggest that upregulated expression of HCN2 (Figure 2 and 3), which has been confirmed the central role in pain signaling, was in accordance with plateaued DNP-like behavioral results (Figure 1). Evidence illustrates the assistance of HCN2 ion channels in increasing forward afferent impulse. Essentially, hyperpolarization below −60 mV activates the membrane-located HCN2 ion channels, which carry depolarized inwards currents (I_*h*_) rebuilding resting membrane potential rapidly [41, 42]. Once coupled with cAMP, enhanced HCN2-I_*h*_ could be obtained, promoting membrane potential to more positive position [14]. A recent study using STZ-treated mice exemplified the dramatically increased cAMP concentration in DRG tissues from pain-evoked diabetic mice than those from control, pain-free diabetic, and even nondiabetic STZ mice [11]. Additional evidence showed selective HCN2 deleted mice with nonenhanced sensitivity to thermal and mechanical stimuli following DN [21]. Together, HCN2 is essential for enablement of pain signaling that fully activated HCN2 channels restore and increased neuronal excitability, and therefore upregulated HCN2 facilitate pain signaling described above. Furthermore, evidence support HCN2-induced repetitive firing could elevate extracellular K^+^ which paradoxically amplify I_*h*_ and promote depolarization [43–45], facilitating the emergence of spontaneous discharge. We have illustrated the dramatical upregulation of HCN2 in DNP rats, highlighting that STZ-induced diabetic DRGs burst out evoked and/or spontaneous afferent signals aggressively.

RETRACTED

Following 7-day riluzole injection (4 mg/kg/d), we observed significantly relieved thermal and mechanical behavior in group riluzole than group DNP and the solvent control (group DMSO), in line with downregulated HCN2 expression (Figures 1–3). Our results support the role of riluzole in alleviating STZ-induced pain-like behaviors potentially via the downregulation of HCN2 expression. Beside, our shortage in lacking per day HCN2 expression following riluzole injection could partially be supported in a recent research of ivabradine, pan-HCN inhibitor, which suggests one single injection can increase diabetic pain thresholds in DN mice, and the benefit could be prolonged by continual administration [11]. Since numerous published studies have included the role of riluzole in diabetes management [46–48], so far, further studies should be recruited to promote understanding of riluzole within diabetes and associated complications administration. Despite paradoxical conditions, we first report riluzole as the alleviator to STZ-induced DNP with the involvement of downregulated HCN2 in lumbar DRG by continual systemic administration in rats.

## 5. Conclusion

Through animal experiments, we explored the effect and possible mechanism of riluzole on DNP. We investigated the change of HCN2 level before and after riluzole treatment in dorsal root ganglion neurons of diabetic neuropathic pain rats. Our results have shown that HCN2 expression was upregulated in DRG tissues of DNP rats, while riluzole downregulated HCN2 expression. Our data suggest riluzole treatments can alleviate pain-like behaviors induced by both thermal and mechanical stimuli in DNP rats under continuous administration; riluzole can treat diabetic neuralgia by downregulating the expression of HCN2 pathway. Riluzole has clinical significance in the treatment of DNP.

## Figures and Tables

**Figure 1:** Effects of riluzole on PWMT and PWTL in DNP rats. (a) Time course of the paw withdrawal thermal latency in STZ-treated rats.  ^*∗*^(*p*) < 0.05 vs. control; #(*p*) < 0.05 vs. DMSO. (b) Time course of sensitivity to mechanical stimuli, shown as the von Frey force threshold for withdrawal, in STZ-treated rats.  ^*∗*^(*p*) < 0.05 vs. control; #(*p*) < 0.05 vs. DMSO.

**Figure 2:** Changes of HCN2 level in DRG detected by western blotting. (a) Western blotting analysis of HCN2 from L3-5 DRG neurons derived of rats in group control, DNP, DMSO, and riluzole. (b) Quantitative analysis showed that riluzole significantly decreased the expression of HCN2 protein in diabetic rats compared to group DMSO.  ^*∗*^(*p*) < 0.05 vs. control; #(*p*) < 0.05 vs. DMSO.

**Figure 3:** Changes of HCN2 level in DRG detected by immunofluorescence analysis. (a) Representative images of the immunofluorescent analysis showing HCN2 (green) expression of L3-5 DRG from control, DNP, DMSO, and riluzole. Scale bar, 100 *μ*m. (b) Quantification of HCN2-positive neurons in the four different groups.  ^*∗*^(*p*) < 0.05 vs. control; #(*p*) < 0.05 vs. DMSO.

## Data Availability

The datasets used and/or analyzed during the current study are available from the corresponding author on reasonable request.
